# Characterizing the Validity of the Inverted Pendulum Model for Quiet Standing

**DOI:** 10.1155/2021/8884614

**Published:** 2021-06-11

**Authors:** Jia-Li Sung, Chih-Yuan Hong, Chin-Hsuan Liu, Posen Lee, Lan-Yuen Guo, Nan-Hung Lin, Chen-Wen Yen, Lih-Jiun Liaw

**Affiliations:** ^1^Department of Mechanical and Electro-Mechanical Engineering, National Sun Yat-Sen University, Kaohsiung 80424, Taiwan; ^2^Department of Occupational Therapy, Kaohsiung Municipal Kai-Syuan Psychiatric Hospital, Kaohsiung 80276, Taiwan; ^3^Department of Occupational Therapy, I-Shou University, Kaohsiung 82445, Taiwan; ^4^Department of Sports Medicine, Kaohsiung Medical University, Kaohsiung 80708, Taiwan; ^5^Department of Physical Therapy, College of Health Science, Kaohsiung Medical University, Kaohsiung 80708, Taiwan; ^6^Neuroscience Research Center, Kaohsiung Medical University, Kaohsiung 80708, Taiwan; ^7^Department of Physical Medicine and Rehabilitation, Kaohsiung Medical University Hospital, Kaohsiung 80708, Taiwan; ^8^Department of Medical Research, Kaohsiung Medical University Hospital, Kaohsiung 80708, Taiwan

## Abstract

By assuming that the human body rotates primarily around the ankle joint in the sagittal plane, the human body has been modelled as a single inverted pendulum (IP) to simulate the human quiet stance. Despite its popularity, the validity of the IP model has been challenged in many studies. Rather than testing the validity of the IP model as a true or false question, this work proposes a feature to quantify the degree of validity of the IP model. The development of the proposed feature is based on the fact that the IP model predicts that the horizontal acceleration of COM is proportional to the COP error which is defined as the difference between the center of pressure (COP) and the vertical projection of the center of mass (COM). Since the horizontal components of the acceleration of COM and the ground reaction force (GRF) are always proportional, the proposed feature is the correlation coefficient between the anterior-posterior (AP) components of GRF and the COP error. The efficacy of the proposed feature is demonstrated by comparing its differences for individuals in two age groups (18–24 and 65–73 years) in quiet standing. The experimental results show that the IP model is more suited for predicting the motion of the older group than the younger group. Our results also show that the proposed feature is more sensitive to aging effects than one of the most reliable and accurate COP-based postural stability features.

## 1. Introduction

With the center of pressure (COP) as the controlling variable and the center of mass (COM) as the controlled variable, the quiet standing human body has been modelled as an inverted pendulum (IP) stabilized by the movement of the ankle joint [1, 2]. An important result of the single joint IP model is that the COM's horizontal acceleration is proportional to the difference between the COP and the vertical projection of the COM. This difference was considered to be the balance control system error signal that induces the COM's horizontal acceleration [1] and will be referred to as the “COP error” hereafter.

The validity of the IP model has been supported by experimental results showing that the COP error is highly linearly correlated with the horizontal acceleration of the COM [2–5]. By representing the human body as an inverted pendulum pivoting about the ankle joint, the ankle strategy employed by the IP model only uses ankle rotations to achieve balance in quiet standing. However, studies that support the multisegment model have found that the motions of nonankle joints are not always negligible. In particular, by directly observing the motion of multiple body joints, several studies have questioned the validity of the single joint IP model by showing that more than one body joint contributes actively and consistently to quiet human stance [6–10].

This work assumes that such inconsistency can at least be partially explained by comparing the relative magnitudes of joint motions. Specifically, if the angular motion of the ankle joint is considerably larger than those of the remaining body joints, it is possible that the IP can still be a satisfactory model for quiet standing posture. In fact, by performing the principal component analysis (PCA) on multiple body joint angles, Pinter et al. [8] discovered that the IP model cannot give a comprehensive description of postural sway data. However, their results also showed that the structure of the first PCA component shows that, in agreement with the prediction of the IP model, the ankle joint displacement gives a good estimate of the COM angle displacement. This result suggests that the validity of the IP model depends on the degree of dominance of the first PCA component. In addition, by identifying that the IP model ignores the ankle-hip coordination, Morasso et al. [11] indicated that the IP model is literally false. However, they also pointed out that if the hip stiffness is sufficiently large, then their multisegment model is practically coincident with the IP model. Morasso et al. [11] also concluded that the IP can still be a practically acceptable model. Since hip stiffness is individually dependent, these results suggest that rather than finding a definite true or false answer for the validity of the IP model, finding a measure that can quantify the degree of validity of the IP model can be valuable.

One of the possible consequences of the inadequacy of the IP model is that the linear proportionality between the COP error and COM's horizontal acceleration may no longer be valid. Based on this observation, this work proposes an index to characterize the degree of validity of the IP model by quantifying the correlation strength between the COP error and horizontal COM acceleration in the anterior-posterior (AP) direction.

Multisegment models should be more competent than the single-segment IP for balance control since they have more biomechanical degrees-of-freedom (DOFs). However, these additional DOFs also imply that the balance control system of the multisegment model needs to be more capable than that of the IP model. As a result, it seems reasonable to assume that, compared to a postural control system that effectively utilizes multiple body joints, a less competent postural control system may lean more toward the IP model since this can reduce the complexity of balance control.

As aging affects the balance control performance during quiet standing [1, 5], this work verified the effectiveness of the proposed feature by using it to differentiate between individuals belonging to two age groups. The assumption is that if the proposed features can outperform the conventional measures used in detecting the effects of aging on postural stability, then the use of the proposed feature as general postural stability measure would warrant further investigation.

By addressing the interactions between the validity of the IP model, the covariation of joint motions, the postural stability, and the proposed feature, it is hoped that the results of this work can increase our understanding of human body segment coordination patterns.

## 2. Methods

### 2.1. Participants

The volunteers participating in this study comprised two age groups: an older age group (68.7 ± 2.96 years, range 65–73 years; BMI 23.9 ± 4.13 kg/m2) and a younger age group (20.1 ± 1.29 years, range 18–24 years; BMI 22.5 ± 3.21 kg/m2). Each group consisted of 10 male and 10 female healthy adults. Based on a self-report and a physical examination, none of the subjects had a pathological condition that would compromise their postural performance. The experimental procedures were approved by the Institutional Review Board of the Kaohsiung Medical University Chung-Ho Memorial Hospital, Kaohsiung, Taiwan.

### 2.2. Measurements

Every subject was tested in two experimental sessions per day for two days. Each session included three 80 s eyes-open-closed trials. In the first 40 s of the trials, the subjects were asked to look straight ahead at a visual reference and stand quietly (with arms at the side) in a comfortable stance near the center of the force platform. By trying to maintain the same posture, the subjects closed their eyes in the remaining 40 s of the trial. The data collected from 5 s to 35 s and 45 s to 75 s of the trials were used for this study. The trials and sessions were separated by approximately one and five minutes of rest, respectively.

The measurement system consisted of a force platform (9286AA, Kistler) connected to a PC-based data acquisition system. The force platform measurements were sampled at 512 Hz with a 14-bit analog-to-digital data acquisition card (USB-6009, National Instruments) connected to a desktop PC. The data processing software was a custom-developed program written in LabVIEW (National Instruments). The signals were filtered by a sixth-order Butterworth filter with a cutoff frequency of 5 Hz.

### 2.3. The Proposed Feature

In the AP direction, the dynamics of the IP model of Figure 1 can be represented by the following equation:

(1) $$\begin{array}{c} x\left(t\right)-p_{x}\left(t\right)=e_{x}\left(t\right)=\frac{I_{a}}{mgh}\ddot{x}\left(t\right)=\frac{I_{a}}{m^{2}gh}{\text{GRF}}_{x}\left(t\right), \end{array}$$

where *x* and *p*_*x*_ are the COM and COP displacements with respect to the ankle joint, respectively, *e*_*x*_ is the COP error, *I*_*a*_ is the mass moment of inertia of the total body about the ankle joint in the sagittal plane, *m* is the mass of the body (excluding the feet), *g* is the acceleration due to gravity, *h* is the COM height above the ankle joint, and GRF_*x*_ is the AP component of the ground reaction force (GRF).

Since the GRF_*x*_ is proportional to the AP component of the COM acceleration, a possible approach to confirm the validity of the IP model is to compute the correlation coefficient between *e*_*x*_ and GRF_*x*_. To compute this coefficient, with COP signal *p*_*x*_ and GRF signal GRF_*x*_ obtained from the force platform, this work uses the zero-point-to-zero-point double integration method to determine the AP component of the COM displacement (i.e., *x* (*t*)) [12]. Specifically, as shown in equation (1), the AP components of COM and COP are equal (i.e., *x* (*t*) = *p*_*x*_ (*t*)) when GRF_*x*_ is equal to zero. By denoting *t*_*i*_ as the *i*th time instant that the value of GRF_*x*_ is equal to zero, we can determine the time response of *x* (*t*) from the following equation via double integration:

(2) $$\begin{array}{c} \;x\left(t\;\right)\;=\;p_{x}\left(t\;\right)+\frac{I_{a}}{m^{2}gh}\;\overset{t}{\underset{t_{i}}{\iint }}{\text{GRF}}_{x}\left(\tau \right)+\;C_{1}\left(t-t_{i}\right)+\;C_{0}, \end{array}$$

for *t*_*i*_ < *t* < *t*_*i*_+1 by determining the integration constants *C*_0_ and *C*_1_ with the boundary conditions *x* (*t*_*i*_) = *p*_*x*_ (*t*_*i*_) and *x* (*t*_*i*+1_) = *p*_*x*_ (*t*_*i*+1_).

The value of the correlation coefficient between *e*_*x*_ and GRF_*x*_ should be close to 1 if the IP model is valid for quiet standing. This work denotes this correlation coefficient as the IP validity index (IPVI) hereafter. Note that a preliminary version of this IPVI measure was proposed in [13]. However, a fundamental problem of that measure is that the COM trajectory was estimated by a heuristic technique. Consequently, the accuracy of the estimated COM trajectory is difficult to verify. This work resolves this problem by using the zero-point-to-zero-point double integration method proposed by [12] to estimate COM. In addition, this work also comprehensively tested the effectiveness of the proposed measure by using IPVI to differentiate between individuals belonging to two age groups.

For comparison, this work also used a COP velocity feature to assess postural stability. Traditionally, the COP velocity can be represented by the mean velocity (MV), mean velocity in the medial-lateral (ML) direction (MV_ML_), and mean velocity in the AP direction (MV_AP_). This study chose MV_AP_ as the benchmark reference since it is considered one of the most sensitive COP measures for postural control assessment [14–16].

### 2.4. Data Analyses

Data analyses were performed to assess the differences between the younger and older groups in the eyes-open condition. The first part of the analysis compared the means of the tested features of the older group to those of the younger group by using independent Student's *t*-tests. For the sake of reliability, this study used the average of the twelve trials (3 measurements/session × 4 sessions) as the sample value.

The second part of the analysis evaluated the association between the proposed feature and postural steadiness quantified by MV_AP_. Specifically, for a given subject, the 30 s process of every experimental trial was first divided into thirty non-overlapping one second windows. This generated 360 windows (12 trials × 30 s) of data for each tested subject. After computing the IPVI and MV_AP_ values for each of these windows, based on the magnitude of IPVI, these windows were divided into two halves. To use the independent Student's *t*-test to assess the differences between the MV_AP_ means of the larger and smaller halves of the IPVI values, this work chose the average MV_AP_ values of each tested subject's larger and smaller halves of the IPVI values as the sample.

To demonstrate the potential of the proposed feature for postural stability assessment, this work used IPVI and MV_AP_ values to classify the two age groups. As noted, there were twelve measurements for each subject. Since the generalization capability of a classifier depends strongly on the training set size, this study used a 3-trial average as the sample to be classified. In particular, by using this 3-trial averaging method, 220 data points were generated for each subject (the number of possible combinations for selecting 3 objects from 12 objects is 220). The 3-trial average method increased the dataset size from 240 (12 measures/person × 20 persons) to 44,000 (220 measures/person × 20 persons) data points for both age groups. Finally, in addition to accuracy, this work also found the area under the curve (AUC) of the receiver operating curve (ROC) since the AUC is considered one of the most effective performance measures for binary classification results [17].

## 3. Results

As shown in Table 1, in agreement with previous studies, the mean value of MV_AP_ of the older group is significantly larger than that of the younger group. Moreover, in agreement with previous studies, the results in Table 1 show that the mean values of the proposed IPVI feature are larger than 0.85 for both age groups. These values of IPVI demonstrate that, in the AP direction, the COP error is highly correlated with the GRF. Table 1 also shows that the mean IPVI value of the older group is significantly larger than that of the younger group. This suggests that the IP model can more accurately represent quiet standing of individuals in the older group than the younger group.

To graphically demonstrate such a relationship, the scatter diagram of the COP error and the horizontal component of COM's acceleration collected from an experimental trial of an older group test subject is depicted in Figure 2. Note that, with a sampling rate of 30 Hz, Figure 2 contains 901 data points. A similar scatter diagram is presented in Figure 3 for a younger group participant. The values of the IPVI feature associated with Figures 2 and 3 are 0.952 and 0.836, respectively. Both Figures 2 and 3 demonstrate a linear relation between COP error and COM's horizontal acceleration. However, with a larger IPVI value, the older group test subject has a more evident linear relation than the younger group test participant.

Table 2 summarizes the comparative results of the MV_AP_ feature associated with the larger and smaller halves of the IPVI values. For both age groups, the mean MV_AP_ of the larger half of the IPVI values is significantly larger than that of the smaller half of the IPVI values.

For the binary classification problem that tries to differentiate the subjects from the two age groups, the resulting AUC and accuracy values are summarized in Table 3. The results show that the proposed feature is more sensitive to the aging-related balance deficits than MV_AP_.

## 4. Discussion

By demonstrating the high correlation of the COP error and GRF signals in the AP direction, the IPVI results in Table 1 support the validity of the IP model. However, since the mean IPVI value of the older group is significantly larger than that of the younger group, the degree of validity of the IP model changes with age. This seems to imply that, by observing the correlation strength between the COP error and the horizontal component of the COM's acceleration, the quiet standing behavior of individuals in the older group is better predicted by an IP model in comparison to the behavior of individuals in the younger group. However, whether aging makes the human body performs more like an inverted pendulum needs to be further verified by observing the actual motions of multiple human body joints.

For both age groups, the results of Table 2 indicate that the mean MV_AP_ of the larger half of the IPVI values is significantly larger than that of the smaller half of the IPVI values. This result and the results of Table 1 show that larger IPVI values are associated with larger MV_AP_ values. As reported by previous studies, large MV_AP_ represents poor postural instability; therefore, it is reasonable to assume that IPVI can also be used to assess postural stability. This assumption is supported by the results of Table 3 showing that IPVI yields larger AUC and higher accuracy than MV_AP_ in classifying the tested subjects of the two age groups. Since MV_AP_ has been considered as one of the most effective COP features for postural stability assessment, the results in Table 3 demonstrate the potential of the proposed feature as a postural stability measure.

The effectiveness of IPVI in characterizing postural stability can be explained as follows. When the human body behaves like an IP, the linear relation between the COP error and COM's horizontal acceleration predicted by equation (1) should be true. As a result, the value of IPVI approaches unity. However, if the human body behaves more like a multisegment system, the linear relation of equation (1) can no longer accurately characterize the interaction between the COP error and COM's horizontal acceleration. By losing such a linear relation, the value of IPVI will decrease from unity and become smaller. With additional biomechanical degrees-of-freedom, multisegment models should be more competent than the single-segment IP model for postural control. Hence, the phenomenon that the value of IPVI decreases from unity implies the employment of a multisegment model which is more capable than the IP model in achieving postural stability.

The fundamental goal of coordinating body joints is to keep the COM within safe limits of the support surface. To achieve this goal, the IP model relies only on ankle motion. In questioning the validity of the IP model, many studies have demonstrated the essential role of other body joints and addressed the importance of joint coordination. For example, by using the uncontrolled manifold (UCM) approach to analyze the effect of joint configuration variance on the stability of the COM, Hsu et al. [7] found that all major joints along the longitudinal axis of the body are equally active during quiet standing. By finding the PCA (principal component analysis) components of the variance of lower leg, upper leg, and head-arms-trunk angles, Pinter [8] discovered the contributions of upper leg and trunk angles to COM motion. By directly measuring ankle, knee, and hip joint kinematics using a vision system, Gunther et al. [9] demonstrated that all leg joints contribute actively to maintaining quiet human stance. These results indicate that the quiet human stance may more appropriately be represented by a multiple degree-of-freedom (DOF) model. Postural control can be formulated as a problem of motor redundancy [18], which occurs when the DOFs of the motor control system are larger than the number of motor control tasks. Such redundancy can be resolved through coupling or constraining the DOFs of the motor control system. This is essentially the strategy employed by the IP model since it uses only the ankle joint to control the COM.

Instead of limiting the functions of the redundant DOFs, the additional DOFs can be used to improve the performance of the motor control tasks or counteract the influences of unwanted disturbances. For example, experimental results have shown that constraining the redundant DOFs by immobilizing the knees, hips, and trunk increased the postural sway [19, 20], whereas including such redundancies can compensate for the effect of breathing on postural steadiness [21].

The results of this study and previous work suggest that the more the redundant DOFs of the balance control system are considered, the less likely the human body behaves like an IP model. In this regard, the proposed IPVI feature represents a simple and effective measure that can relate the degree of validity of the IP model with the coordination pattern of the body joints. By monitoring the joint motion with vision systems, a promising future direction is to study the interactions between joint coordination patterns, postural stability, and the proposed feature.

## 5. Conclusions

This paper introduces a feature to characterize the degree of validity of the inverted pendulum (IP) model for a quiet standing human body. The proposed feature quantifies the correlation strength between the COP error (the difference between the COP and the vertical projection of COM) and the AP component of the ground reaction force (GRF_*x*_). By comparing the proposed IP validity index (IPVI) values of individuals in two age groups, it is found that the IP model can more accurately predict the correlation strength between the COP error and GRF*x* of the older group than the younger group. This result seems to suggest that the IP model is better at characterizing and predicting the motion of individuals in the older group than the younger group. Furthermore, the results of this work support previous studies that demonstrate the active role of multiple body joints on postural balance. This suggests that the redundant DOFs of the body joints can be used in more advanced models to represent postural dynamics, while diminishing the validity of the IP model. As a validity index of the IP model, the proposed feature can be useful to assess the quiet standing coordination patterns of the body segments. Experimental results demonstrate the potential of the proposed feature for assessing postural stability.

## Figures and Tables

**Figure 1:** Inverted pendulum model for standing.

**Figure 2:** The scatter diagram of the COP error and COM's horizontal acceleration for an older group test subject. The corresponding correlation coefficient value is 0.952.

**Figure 3:** The scatter diagram of the COP error and COM's horizontal acceleration for a younger group test subject. The corresponding correlation coefficient value is 0.836.

**Table 1:** Mean, standard deviation, and *p* values of the COP feature MVAP and the proposed feature IPVI.

Features	Age group		*p* values
	Younger	Older	
MV_AP_	5.45 ± 1.06	7.28 ± 2.00	9.52 × 10^−4^
IPVI	0.869 ± 0.024	0.919 ± 0.017	6.83 × 10^−9^

Values of the features are mean ± standard deviation. Units of features are as follows: mm/s (MV_AP_) and dimensionless (IPVI).

**Table 2:** Mean, standard deviation, and *p* values of the COP feature MVAP for the larger and smaller halves of the IPVI feature values.

Age group	IPVI values		*p* values
	The larger half	The smaller half	
Younger	6.06 ± 0.70	4.84 ± 0.83	2.25 × 10^−3^
Older	8.87 ± 1.55	5.78 ± 1.00	1.00 × 10^−5^

Values of the features are mean ± standard deviation. Unit of MV_AP_ is mm/s.

**Table 3:** Accuracy and AUC for the COP feature MVAP and the proposed feature IPVI.

Features	AUC	Accuracy
IPVI	0.933	0.849
MV_AP_	0.778	0.733

## Data Availability

The clinical data used to support the findings of this study have not been made available because of the protection of patient privacy.
